This article has been retracted.

# Health risk assessment of heavy metals via consumption of dietary vegetables using wastewater for irrigation in Swabi, Khyber Pakhtunkhwa, Pakistan

**DOI:** 10.1371/journal.pone.0255853

**Published:** 2021-08-11

**Authors:** Fawad Ali, Muhammad Israr, Shafiq Ur Rehman, Azizullah Azizullah, Hussain Gulab, Muhammad Idrees, Rashid Iqbal, Aishma Khattak, Majid Hussain, Fahad Mohammed Al-Zuaibr

**Affiliations:** 1 Department of Chemistry, Bacha Khan University Charsadda, Charsadda, Khyber Pakhtunkhwa, Pakistan; 2 Department of Biology, The University of Haripur, Haripur, Khyber Pakhtunkhwa, Pakistan; 3 College of Life Science, Hebei Normal University, Shijiazhuang, Hebei, PR China; 4 Department of Biotechnology, University of Swabi, Swabi, Khyber Pakhtunkhwa, Pakistan; 5 Department of Agronomy, Faculty of Agriculture and Environment, Islamia University, Bahawalpur, Pakistan; 6 Department of Bioinformatics, Benazir Bhutto Women University Peshawar, Khyber Pakhtunkhwa, Pakistan; 7 Department of Forest and Wildlife Management, University of Haripur, Haripur City, Khyber Pakhtunkhwa, Pakistan; 8 Department of Biology, Faculty of Science, University of Tabuk, Tabuk, Saudi Arabia; Ghazi University, PAKISTAN

## Abstract

Health assumptions to the population due to the utilization of contaminated vegetables have been a great concern all over the world. In this study, an investigation has been conducted to ascertain metal concentrations in the wastewater, soil and commonly consumed vegetables from the vicinity of Gadoon Industrial Estate Swabi, Khyber Pakhtunkhwa Pakistan. Physicochemical parameters such as pH, electrical conductivity (EC), total dissolved solids (TDS), total suspended solids (TSS) and total solids (TS) and heavy metals such as Pb, Cr, Cd, Ni, Zn, Cu, Fe, Mn were determined using Atomic Absorption Spectrophotometer (AAS). Moreover, possible health risks due to the consumption of vegetables have also been estimated. pH and TSS in wastewater were found to be higher than the permissible limit set by WHO (1996). These results revealed that Cr concentration in the wastewater was above the permissible limits of United States Environmental Protection Agency (USEPA) which may lead to a detrimental effect on soil quality deterioration, ultimately leading to food contamination. ANOVA analysis demonstrated a significant difference in soil samples for Pb, Cr, Cd, Ni, Zn and Cu at p ≤ 0.001, for Mn at p ≤ 0.05 while no significant difference was observed for Fe respectively. ANOVA analysis also exhibited the highest mean value for Pb, Cr, Cd and Zn in vegetables. A substantial positive correlation was found among the soil and vegetable contamination. The transfer factor for Cr, Pb, Zn, Mn, Ni, Cd and Cu was greater than 0.5 due to contamination caused by domestic discharges and industrial effluents. Health assessment via consumption of dietary vegetables revealed a higher level than the permissible limit (HRI > 1) for Pb and Cd in children and adults. Enrichment factor (EF) due to consumption of vegetables was found higher for Pb and Cr respectively. Based on the findings of this study, there would be a significant risk to the consumers associated with consumptions of vegetables being cultivated in Gadoon Industrial Estate area of district Swabi. Therefore, strict regulatory control measures are highly recommended for the safety of vegetables originated from the study area.

## Introduction

Life on earth depends on the availability of a sufficient amount of freshwater. The estimated quantity of water on earth is about 1.4 trillion cubic meters [1]. Agriculture is mainly based upon two natural resources i.e. soil and water, deficiency in any of them will pose a threat to productivity. The cultivated land is 12.49 million hectares of the total 20.63 million hectares of land in Pakistan, of which nearly 2.54 hectares area is used for the cultivation of vegetables [2]. One estimate shows that about 20 million hectares of area in around 50 countries uses wastewater for agricultural activities and it will further enhance in near future [3–6]. Heavy metals are generally considered to be elements having metallic characteristics like ductility, conductivity, etc. and with an atomic number of more than 20. Various pollutants are responsible for damages to the ecosystem but heavy metals have much importance in terms of environmental contamination [7]. In all contaminants, heavy metals are the main contributing pollutants because of altering the physical and chemical properties of the ecosystem [8]. The toxic level of heavy metals is not necessarily due to high exposure because uptake of heavy metals takes place continuously, crossing the permissible range in most of the cases [9].

Heavy metals, also known as the trace elements of the periodic table, are very important in the water reservoir and water pollution due to their non-biodegradable nature [10]. These heavy metals on the other hand are also very important for the proper functioning of biological systems. But the high level of trace metals in water reservoirs causes various threats to plants, animals and human life. The issue is due to the transfer of these metals from water to soil and then to vegetables [11]. Heavy metals have a density of more than 5 g/cm^3^ which is five times more compared to water. There are about 38 heavy metals in the periodic table but only 12 of them are important for human health’s which are Cu, Ni, Fe, Zn, Mo, Co, Mn, Cd, Cr, Sn, Hg and Pb [12]. Of all these, toxic metals having specific gravity 5 times more than water are As (5.7 g/cm^3^), Cd (8.65 g/cm^3^), Fe (7.9 g/cm^3^), Pb (11.34 g/cm^3^) and Hg (13.546 g/cm^3^) [13]. In the case of health, various heavy metals are responsible for causing diseases but important of them are lead and cadmium [14]. Toxic levels of all essential and nonessential trace metals change the three-dimensional structure of an enzyme, destroy cell membrane and alter cellular functions [15]. Toxicity due to trace metals is a matter of great concern throughout the globe because of its carcinogenic and neurotoxic effects [16]. Heavy metals intake in humans is associated with blood acidity, cancer, kidney problems, growth retardation and ultimately death. With this in mind, the present study was conducted to investigate the concentration level of selected heavy metals in selected vegetables, soil and wastewater samples collected from Gadoon Industrial Estate, Swabi Khyber Pakhtunkhwa Pakistan, where the canals used for irrigation purposes are highly contaminated with heavy metals being released from various industries in the area. In this regard, we have also investigated the possible health risk associated with dietary exposure to these potentially toxic metals by calculating the Health Risk Index (HRI).

## Materials and methods

### Geographical location of the study area

Swabi is the fourth popular district of Khyber Pakhtunkhwa, Pakistan. It was part of district Peshawar and later on a subdivision of Mardan and finally become an independent district in 1988. Swabi is bounded on the east by Haripur, on the north by Buner, on the south by Attock and West by Nowshera and Mardan. It is situated among rivers Kabul and Indus. It has an area of 1,543 km^2^ having a population of 1.8 million. It is located at 34.1442° N, 72.3785° E of Khyber Pakhtunkhwa, Pakistan. Swabi remained part of the Gandhara civilization and hund which were one of the most important capitals of Hindu Shahi. The great Alexander crossed the Indus River through Swabi. The people of Swabi are called Swabval. The climate of Swabi is warm and temperate. There was much precipitation in summer as compared to winter. The annual mean temperature and rainfall recorded in Swabi was 22.2°C was 639 mm [17].

### Sampling

Farming fields were selected in the vicinity of Gadoon Industrial Estate Swabi. Various industries such as leather, metals processing, paper mills, ghee, dyeing, battery manufacturing, pharmaceuticals and nestle, etc. were present near the selected fields. Based on the geologic and tectonic analysis, Swabi was divided into two regions, one main region (sector-S) and the other control area (sector-SC). Both regions further have 21 microsites in the study area. A total of 42 microsites were selected from Swabi. Distance between Swabi (sector-S) and control area (sector-SC) was about 20 km (Fig 1).

**Fig 1:** Map of sampling area.

All samples of water, soil and dietary vegetables were collected from these selected fields. All equipment and glassware were soaked with 30% HNO_3_ and placed for 24 h, afterward rinsed with double deionized water before used for analysis.

### Water samples collection and preparation

Water samples (500 mL) were collected in the plastic bottle using a vinyl glove from different areas of each selected site during January 2020 to December 2020. The empty plastic bottles were the first acid washed with 5% HNO_3_ to avoid contamination and then rinsed with double deionized water. About 50 samples of wastewater were collected from different selected sectors, which are used for irrigation of dietary vegetables. Some important parameters like pH, Electrical Conductivity were measured on the spot. The samples were directly transported to the laboratory and about 1 mL of concentrated HNO_3_ was added into samples to avoid any kind of microbial growth.

### Water samples digestion

Water samples (50 mL) both clean and untreated wastewater were digested using 10 mL concentrated HNO_3_ at 80°C on a hot plate for about 60 min until a transparent solution formed. After digestion, the samples were filtered with Whatman No.42 filter paper and the filtrate were diluted to about 50 mL with distilled water. Heavy metals were determined by using double beam Perkin Elmer Atomic Absorption Spectrometer Model 2380 (USA) having graphite furnace, pyro-coated graphite tube and autosampler. Radiation source such as hollow cathode lamp was used. The Pb, Cr, Cd and Ni were analyzed by electrothermal atomic absorption spectrometer while Cu and Zn were determined by Flame Absorption Spectrometer [18].

### Soil samples collection and preparation

Soil composite samples (1 kg) using vinyl gloves were collected from twenty-eight agricultural fields of both wastewater and clean water irrigated sites of main and control sectors. Control sectors were selected few kilometers away from urban areas having low traffic density, less human and industrial activities. Soil samples were collected in triplicate randomly at the same time from different areas of top layers (0–30 cm) manually through a spiral auger or plastic scooper. The top layer was considered essential due to involvement in biological activities and all interconversions take place between soil and water in this layer. Samples were air-dried, crushed, passed through 2 mm mesh and stored at ambient temperature in tightly packed zip plastic bag or Kraft paper envelops, carried to the laboratory and kept in desiccators until digestion and analysis.

### Soil samples digestion

Soil samples were digested in Teflon beakers by taking 1g soil with 15 mL tri acid mixture of HNO_3,_ HClO_4_ and H_2_SO_4_ at a 5:1:1 ratio at a temperature of 100°C. The mixture was heated until a clear solution was formed. After cooling, the digested sample was filtered using Whatman No. 42 filter paper and the volume of the filtrate was made 50 mL by adding double de-ionized water. The filtrate was then analyzed for heavy metals i.e. Pb, Cr, Cd, Ni, Zn, Cu, Fe and Mn by using AAS in air acetylene flame mode [19]. The suspension was filtered through Whatman No. 42 filter paper. pH and EC were assayed through digital Cole Parmer 5983 pH meter and EC meter InoLab model E 163694 at room temperature.

### Vegetable samples collection and preparation

Dietary vegetables were randomly collected from the same sector from where soil and untreated wastewater were taken. Description of vegetables along with local and botanical names are listed in S1 Table. These vegetables were cultivated for home consumption and sale to the local population of Swabi. A total of 50 samples were taken for each vegetable in plastic bags. About 1 kg sample of every vegetable was taken and transported to the laboratory and was stored in ambient condition for analysis. Edible parts of the vegetables were rinsed with clean water to remove any soil particles using a vinyl brush. Extra water was removed using blotting paper, samples were then cut into pieces, air-dried and then oven-dried at 80°C until constant weight was achieved. The oven-dried samples were made powdered using a steel grinder and sieved through 2 mm mesh and were stored at ambient temperature for digestion.

### Vegetable samples digestion

A dried vegetable sample (0.5 g) was taken in a Pyrex beaker. About 15 mL of acid mixture HNO_3,_ HClO_4_ and H_2_SO_4_ (5:1:1) ratio was added to the beaker and placed overnight without heating. Afterward, digestion tubes were put at a temperature of 80°C for 60 min and then the temperature was gradually increased to 120–130°C until a clear solution was obtained. The samples were filtered when digestion was completed and the volume was made 50 mL by adding double de-ionized water. A blank solution was also run following the same procedure without adding the sample. The digested vegetable samples were analyzed for micronutrients (Fe, Zn, Mn, Cu) and toxic elements (Ni, Cd, Cr, Pb) using Atomic Absorption Spectrophotometer (AAS, Perkin-Elmer 2380 USA). A specific hollow cathode lamp was used for each metal. Air acetylene flame was used as a fuel source [20].

### Physicochemical parameters

The collected water samples were analyzed for pH and electrical conductivity (EC) at the spot through digital Cole Parmer 5983 pH meter and EC meter InoLab model E 163694 at room temperature. Total dissolved solids (TDS), total suspended solids (TSS) and total solids (TS) were measured in mg/L using a Consort Electrochemical Analyzer.

### Standard stock solutions

Standard stock solutions (1000 mg/L) were prepared for each metal, for Pb added 1.5 g of Pb(NO_3_)_2_ in 250 mLvolumetric flask, for Cr added 3.8 g of Potassium dichromate in 200 mL volumetric flask, for Ni added 1 g in 10 mL of HNO_3_, for Zn dissolved 100 mg in 25 mL of hydrochloric acid, for Cu dissovled 1 g in 25 mL of HNO_3_, for Fe dissolved 1 g in 10 mL of HCl, then added all these in a 1-liter flask and diluted it by adding double deionized water. The different working standard solution was prepared for the analysis (25, 50, 100 mg/L). The instrument was calibrated under standard conditions and heavy metals were determined using an autosampler (Table 1).

**Table 1:** Analytical conditions for the determination of heavy metals in water using graphite furnace.

Parameter	Pb	Cr	Cd	Ni	Zn	Cu	Fe	Mn
Wavelength	283.3nm	357.9nm	228.8	232nm	213.9nm	325.8nm	248.3nm	279.5
Mode	Abs	Abs	Abs	Abs	Abs	Abs	Abs	Abs
Slit width	0.7nm	0.7nm	0.7nm	0.2nm	0.7nm	0.7nm	0.2nm	0.2nm
Tube/site	Pyro/Platform	Pyro/Platform	Pyro/Platform	Pyro/Platform	Pyro/Platform	Pyro/Platform	Pyro/Platform	Pyro/Platform
Matrix modifier	0.05mg H_4_H_2_PO_4_	0.05mg (NO_3_)_2_	Nil	0.05mg (NO_3_)_2_	0.05mg H_4_H_2_PO_4_	Nil	0.05mg (NO_3_)_2_	Nil
Pretreated T°C	1200	1600	Nil	1400	1200	1200	1400	Nil
Acetylene (L/min)	2.0	2.5	2.0	2.0	2.0	2.0	2.0	2.0
Air (L/min)	17	17	17	17	17	17	17	17
Lamp current (Ma)	30	25	4	25	15	15	15	20
Atomization T°C	2300	2500	Nil	2500	2300	2300	2400	Nil
Detection limit	0.05	0.004	Nil	0.07	0.02	0.014	5	Nil

### Transfer factor (TF)

Toxic metal concentrations were determined in extracts of soil and vegetables on a dry weight premise. Then metal to vegetable transfer was calculated by using the formula [21];

$$TF=\frac{C_{Vegetable}}{C_{Soil}}$$

Where C _vegetable_ is the concentration of heavy metal in vegetables and C _soil_ is the concentration in soil.

### Daily intake of metals (DIM)

The normal daily intake of vegetables in adults and children was obtained during the study through a survey. The daily intakes of metals were determined by mathematical relation [18];

$$DIM=\frac{C_{metals}\times C_{factor}\times D_{food\;intake}}{B_{average\;weight}}.$$

Where C _metal_, C _factor_, D _food intake_ and B _average weight_ indicate toxic metal uptake in vegetables, transformation element (0.085), daily intake of vegetable and average body weight, respectively.

Both male and female adults (18–60 years) and children (7–17 years) were considered in the poll review. The normal weight for adults and children’s body in Pakistan was proposed to be 60 kg and 35 kg respectively.

### Health risk index (HRI)

The health risk index was figured as the proportion of assessed presentation of test harvests and oral reference measurement [18]. The HRI ˃ 1 will be considered as the exposed population is not safe [22].


$$HRI=\frac{DIM}{RFD}$$

Where DIM is a daily intake of metals and RFD is an oral reference dose.

### Enrichment factor (EF)

Enrichment factor was used to examine the transfer of toxic metals from soil to eatable bits of vegetables and it will also show differences in metal fixations in vegetables between the different localities.

EF was ascertained by the formula [23];

$$EF=\frac{Concentration\;of\;metal\;in\;edible\;part\;at\;WWI\;site-Concentration\;of\;metal\;in\;soil\;at\;WWI\;site}{Concentration\;of\;metal\;in\;edible\;part\;at\;CWI\;site/Concentration\;of\;metal\;in\;soil\;at\;CWI\;site}$$

Where WWI is a wastewater irrigated site while CWI is clean water irrigated site.

## Results and discussions

### Physicochemical and heavy metals concentration in wastewater

Table 2 shows the physicochemical parameters of water collected from both fresh and wastewater areas. The pH of wastewater ranged from 7.4–9.4 with a mean ± SD of 8.4 ± 0.64 in sector-S. In the less polluted sector SC, pH ranged from 7.3–8.0 with a mean ± SD value of 7.9 ± 0.48 respectively. A pH of wastewater showed alkaline nature due to industrial effluents as given by WHO (6.5–8.5). Electrical conductivity (EC) ranged from 1.1–2.3 dS/m with an average ± SD of 1.5 ± 0.37, in sector-S. EC value in less polluted sector SC ranged from 1.1–1.6 dS/m with mean ± SD of 1.2 ± 0.13 respectively. In sector S, TS ranged between 850–1160 mg/L, mean ± SD of 1020 ± 109.7, TDS between 390–620 mg/L, mean ± SD 547.8 ± 65.88 and TSS ranged between 340–465 mg/L, mean ± SD 393 ± 42.8, respectively while in less polluted sector SC, these values ranged from 800–1000 mg/L, mean ± SD 907 ± 69.49, 340–600 mg/L mean ± SD 472 ± 86.82 and 310–430 mg/L mean ± SD 370 ± 42.24, respectively. TS of the wastewater was found to cross the permissible limit of WHO (1000 mg/L). Industries in the near locality mainly dispose of various pollutants which ultimately increase EC and the previous study reported that pH and EC of discharges were related to the type of chemicals used by factories and also to the types of industries [24].

**Table 2:** Descriptive statistics for physicochemical properties and heavy metals concentration in water of Swabi.

	Sector S (wastewater)				Sector SC (wastewater)					
	Min	Max	Mean ± SD	Range	CV	Min	Max	Mean ± SD	Range	CV
**pH**	7.40	9.40	8.42±0.64	2.00	0.41	7.30	8.90	7.96±0.48	1.60	0.23
**EC (dSm** ^**-1**^ **)**	1.10	2.30	1.50±0.37	1.20	0.14	1.10	1.60	1.28±0.13	0.50	0.02
**TS (mgL** ^**-1**^ **)**	740	1085	940±94.91	345	9008	680	940	842±78.23	260	6121
**TSS (mgL** ^**-1**^ **)**	340	465	393±42.83	125	1835	310	430	370±42.24	120	1784
**TDS (mgL** ^**-1**^ **)**	390	620	547±65.88	230	4340	340	600	472±86.82	260	7539
**Pb (mg L** ^**-1**^ **)**	0.57	1.14	0.79±0.18	0.57	0.03	0.10	0.35	0.22±0.06	0.25	0.004
**Cr (mg L** ^**-1**^ **)**	4.02	12.99	8.04±2.41	8.96	5.82	1.01	3.33	2.08±0.71	2.31	0.50
**Cd (mg L** ^**-1**^ **)**	0.02	0.03	0.02±0.002	0.01	0.00	0.02	0.02	0.01±0.001	0.00	0.00
**Ni (mg L** ^**-1**^ **)**	0.31	0.60	0.46±0.11	0.28	0.01	0.21	0.37	0.29±0.05	0.16	0.003
**Zn (mg L** ^**-1**^ **)**	0.16	0.19	0.17±0.008	0.03	0.00	0.15	0.17	0.15±0.005	0.02	0.00
**Cu (mg L** ^**-1**^ **)**	0.08	0.25	0.14±0.04	0.17	0.002	0.04	0.14	0.08±0.03	0.10	0.001
**Fe (mg L** ^**-1**^ **)**	0.51	0.82	0.68±0.09	0.32	0.008	0.32	0.45	0.38±0.04	0.14	0.002
**Mn (mg L** ^**-1**^ **)**	0.15	0.55	0.32±0.09	0.40	0.01	0.10	0.35	0.24±0.06	0.25	0.005

Max stands for maximum, Min for minimum, SD Standard deviation.

The concentration of Pb, Cr, Cd, Ni, Zn, Cu, Fe and Mn in wastewater ranged from 0.569–1.135, 4.023–12.985, 0.020–0.028, 0.314–0.595, 0.160–0.185, 0.08–0.25, 0.505–0.821, 0.15–0.55 mg/L, while in freshwater were 0.103–0.350, 1.012–3.326, 0.016–0.020, 0.210–0.370, 0.150–0.168, 0.04–0.14, 0.315–0.450 and 0.10–0.55 mg/L, respectively. ANOVA analysis showed a significant difference for Fe and Mn at p ≤ 0.05 while Pb, Cr, Cd, Ni, Zn and Cu were at p ≤ 0.01 between wastewater and freshwater. Farid investigated a high concentration of Cr in wastewater which was posing threat to human consumption in Faisalabad, Pakistan [25]. Kachenko and Singh analyzed Cd concentration in wastewater samples at Boolaroo, Australia which was much lower compared to the current study [26].

### Heavy metals concentration in soil

The concentration of Pb, Cr, Cd, Ni, Zn, Cu, Fe and Mn in wastewater irrigated soil ranged from 4.17–7.34, 0.34–0.96, 0.25–0.81, 2.12–4.35, 1.25–2.62, 6.5–11.5, 10.5–16.5, 1.01–2.25 mg/kg, while in freshwater irrigated soil were 2.25–4.35, 0.20–0.55, 0.20–0.50, 1.05–3.00, 1.00–1.90, 3.00–5.00, 6.00–9.50, 0.80–1.00 respectively (Table 3). Decreasing order of heavy metals in the soil of sectors, S and SC were Fe > Cu > Zn > Ni > Mn > Pb > Cr > Cd and Fe > Mn > Ni > Cu > Zn > Pb > Cr = Cd mg/kg respectively. The application of wastewater for irrigation purposes in the vicinity of tanneries accumulates a greater amount of Cr in soil and vegetables [27]. Liu *et al*. determined Ni concentration in wastewater irrigating soil in Zhengzhou city of China [28], which was much less than the present study of Khyber Pakhtunkhwa, Province, Pakistan. ANOVA analysis showed a significant difference for Mn at p ≤ 0.05, Pb, Cr, Cd, Ni, Zn and Cu were significantly different at p ≤ 0.01 between wastewater and fresh irrigating soil respectively (Table 4).

**Table 3:** Descriptive statistics for physicochemical properties and heavy metals concentration in soil of Swabi.

	Sector S (wastewater irrigated soil)				Sector SC (wastewater irrigated soil)					
	Min	Max	Mean ± SD	Range	CV	Min	Max	Mean ± SD	Range	CV
**Pb (mg kg** ^**-1**^ **)**	4.17	7.34	5.68±0.94	3.17	0.89	2.25	4.35	3.01±0.73	2.10	0.54
**Cr (mg kg** ^**-1**^ **)**	0.34	0.96	0.58±0.20	0.62	0.04	0.20	0.55	0.33±0.13	0.35	0.02
**Cd (mg kg** ^**-1**^ **)**	0.25	0.81	0.50±0.20	0.56	0.04	0.20	0.50	0.33±0.11	0.30	0.01
**Ni (mg kg** ^**-1**^ **)**	13	25	17.85±3.21	12	10.32	9.50	20	14.9±2.86	10.50	8.20
**Zn (mg kg** ^**-1**^ **)**	10.50	24	18.30±4.71	13.50	22.21	8.50	19	13.4±3.16	10.50	10.02
**Cu (mg kg** ^**-1**^ **)**	10	24	18.57±3.99	14	15.93	10	24	13.9±3.32	14	11.08
**Fe (mg kg** ^**-1**^ **)**	12.50	35.50	22.59±8.54	23	73.07	10.50	30.50	19.5±6.84	20	46.81
**Mn (mg kg** ^**-1**^ **)**	12.11	22.45	17.14±3.56	10.34	12.69	11.11	19.45	16.5±2.62	8.34	6.91

Max stands for maximum, Min for minimum, SD for standard deviation.

**Table 4:** ANOVA analysis for heavy metals in water and soil of two different sectors in Swabi.

Water								
Sectors	Pb	Cr	Cd	Ni	Zn	Cu	Fe	Mn
**Sector-S (wastewater)**	0.79 a	8.04 a	0.02 a	0.46 a	0.17 a	0.14 a	0.68 a	0.32 a
**Sector-SC (wastewater)**	0.22 b	2.08 b	0.02 b	0.29 b	0.16 b	0.09 b	0.38 b	0.25 b
**Significant**	**	**	**	**	**	**	*	*
**Soil**								
**Sectors**	Pb	Cr	Cd	Ni	Zn	Cu	Fe	Mn
**Sector-S (soil)**	5.68 a	0.58 a	0.50 a	17.85 a	18.30 a	18.57 a	22.59 a	17.14 a
**Sector-SC (soil)**	3.01b	0.33 b	0.33 b	14.92 b	13.04 b	13.92 b	19.35 a	16.15 b
**Significant**	**	**	**	**	**	**	Ns	*

Letters a, b, show significant differences

*stands for significant at 0.05

**for significant at 0.01, ns for not significant.

### Heavy metals in wastewater irrigated vegetables

The concentrations of Pb, Cr, Cd, Ni, Zn, Cu, Fe and Mn in spinach, cabbage, cauliflower, radish, turnip, tinda, carrot, lettuce, colocasia, bootle gourd, tomato, cucumber, potato, red pepper, coriander, bitter gourd, green pepper, brinjal, pea, pumpkin, onion, garlic, green amaranth in wastewater irrigated sectors ranged from 0.70–18.14, 0.13–17, 0.02–3.64, 0.02–26.85, 0.04–95.83, 0.05–25.83, 7.42–102.14, 7.03–44.16 mg/kg while in freshwater areas, 0.39–4.42, 0.14–4.43, 0.02–2.57, 0.02–18.85, 0.03–75, 0.03–19.5, 4.69–53.66, 3.84–32.14 mg/kg respectively as shown in Figs 2 and 3.

**Fig 2:** Heavy metals concentration in vegetables of sector-S.

**Fig 3:** Heavy metals concentration in vegetables of sector-SC.

Concentrations of Pb, Cr and Cd were found higher than the permissible limit of WHO (1996) in most of the study areas.

The current investigation showed accumulation of Pb, Cr, Cd and Ni in wastewater irrigating vegetables. In most vegetables, these metals crossed permissible limits of WHO (1996). Khanna also reported a high concentration of heavy metals in wastewater irrigating vegetables [9]. A consistent findings was reported by Sajida *et al*. They investigated heavy metal accumulation in wastewater irrigated vegetables posing threat to human’s health in Peshawar, KP Pakistan [29].

### Heavy metals transfer factor from soil to vegetables (TF)

Table 5 shows the mean value of transfer factor for heavy metals like Pb, Cr, Cd, Ni, Zn, Cu, Fe and Mn in sector-S ranged from 0.06–3.56, 0.18–23.48, 0.02–3.98, 0.01–15.38, 0.008–7.27, 0.005–5, 0.54–9.64 and 1.45–26.9. The decreasing order of TF of sector-S was Cr > Zn > Ni > Fe > Cd > Mn > Pb > Cu. The mean value of transfer factor for heavy metals like Pb, Cr, Cd, Ni, Zn, Cu, Fe and Mn in sector-SC ranged from 0.03–2.93, 0.52–19.62, 0.05–6.95, 0.05–40.35, 0.01–35.9, 0.008–7.66, 0.47–29.73 and 1.88–34.5 respectively (Table 5). The decreasing order of TF of sector-SC was Cr > Cd > Zn > Fe > Mn > Cu > Ni > Pb. The present study showed a higher value of TF for Pb, Cr, Cd, Zn and Fe as indicated by previous researchers [21, 28]. TF mainly depends on soil properties and metal concentrations. Higher TF in leafy vegetables was due to high transpiration rate and more surface area of leaves. Low TF value was due to more retention of metals in soil. Some researchers also showed various patterns of TF both in clean water and wastewater irrigation [21, 28].

**Table 5:** Heavy metals transfer factor for vegetables grown in Swabi.

Vegetables	Sector	Pb	Cr	Cd	Ni	Zn	Cu	Fe	Mn
**Spinach**	S	1.34	9.20	0.89	5.09	0.88	0.82	0.56	2.37
	SC	0.99	10.85	2.35	1.19	1.18	1.07	0.53	1.99
**Cabbage**	S	2.38	9.75	2.82	1.07	0.77	0.96	0.84	0.54
	SC	0.99	9.27	2.92	0.99	0.92	1.01	0.82	0.48
**Cauliflower**	S	2.12	16.34	0.71	0.93	0.5	0.95	0.72	0.99
	SC	0.81	11.07	1.37	0.93	0.43	0.67	0.69	0.97
**Radish**	S	0.46	0.74	0.70	0.07	0.08	0.52	0.55	0.41
	SC	0.38	0.28	0.75	0.03	0.08	0.63	0.24	0.23
**Turnip**	S	0.76	4.80	1.89	0.88	0.77	0.44	0.32	1.58
	SC	0.48	5.25	5.32	0.77	0.84	0.30	0.37	1.32
**Tinda**	S	0.31	2.41	0.90	0.92	0.72	0.31	0.70	1.08
	SC	0.35	6.05	2.85	0.84	0.89	0.34	0.59	0.88
**Carrot**	S	1.06	5.83	1	0.91	0.48	0.83	1.16	1.43
	SC	0.84	7.85	3.42	1.06	0.60	0.93	0.93	0.96
**Lettuce**	S	0.67	5.14	2.34	1.50	0.80	0.55	0.83	1.54
	SC	1.03	8.02	6.42	1.23	0.93	0.37	0.45	1.13
**Colocasia**	S	0.34	2	1.09	1.28	0.40	1.03	0.51	1.31
	SC	0.49	4.90	3.37	1.26	0.46	0.80	0.37	0.96
**Bootle gourd**	S	0.09	0.72	0.03	0.36	1.14	0.54	0.93	0.99
	SC	0.12	1.25	0.05	0.25	1.01	0.56	0.84	0.99
**Tomato**	S	0.13	0.94	0.01	0.001	1.19	1.30	2.81	0.50
	SC	0.20	1.80	0.05	0.001	1.41	1.12	1.69	0.45
**Cucumber**	S	0.18	1.16	0.59	0.78	2.05	0.62	4.51	0.89
	SC	0.27	1.62	0.92	0.82	2.30	0.53	2.65	0.79
**Potato**	S	0.33	0.60	0.38	0.16	1.15	0.43	0.53	1.05
	SC	0.42	1.47	1.02	0.18	1.53	0.58	0.61	1.08
**Red pepper**	S	0.13	0.50	0.01	0.01	1.25	1.39	3.17	1.45
	SC	0.18	1.10	0.07	0.01	1.65	1.40	2.77	1.14
**Coriander**	S	0.14	0.64	0.11	0.56	1.38	0.83	4.42	1.28
	SC	0.16	1.17	0.20	0.30	1.53	0.92	2.62	1.12
**Bitter gourd**	S	0.13	0.12	0.02	0.002	0.002	0.002	1	0.58
	SC	0.15	0.50	0.05	0.002	0.002	0.002	1.04	0.43
**Green pepper**	S	0.11	0.20	0.21	0.46	5.27	0.70	4.20	2.57
	SC	0.13	0.35	0.27	0.45	5.76	0.79	3.83	1.95
**Brinjal**	S	0.12	0.72	0.14	0.15	1.05	1.30	3.10	2.09
	SC	0.16	1.85	0.35	0.15	1.07	1.29	2.54	1.80
**Pea**	S	0.57	1.53	1.72	1.16	1.31	0.11	1	2.28
	SC	0.42	2.95	1.30	1.22	1.43	0.09	0.76	1.14
**Pumpkin**	S	0.06	1.25	0.02	0.48	1.94	0.93	0.88	1.23
	SC	0.09	1.7	0.05	0.32	2.23	1.14	1.01	1.16
**Onion**	S	0.53	1.60	1.20	0.87	1.03	0.03	0.70	0.74
	SC	0.29	1.7	1.52	0.81	1.08	0.04	0.58	0.62
**Garlic**	S	0.66	1.49	1.62	1.26	1.89	0.33	1.23	1.32
	SC	0.54	2.37	3.1	0.93	2.49	0.29	1.16	1.04
**Green amaranth**	S	0.27	0.88	0.12	0.13	2.02	0.58	0.61	1.35
	SC	0.34	2.27	0.35	0.11	2.82	0.59	0.69	1.13

### Daily intake of metals and health risk index for vegetables

The daily intake of metal value was high for vegetables using wastewater irrigated soil compared to tubewell irrigated soil. Vegetables grew in contaminated soil result in health risks of metals consumption in comparison to uncontaminated soil. The daily intake of metals in Swabi for Pb, Cr, Cd, Ni, Zn, Cu, Fe and Mn for adults ranged from 2.64E-04 to 9.79E-03, 7.02E-05 to 9.18E-03, 1.08E-05 to 1.96E-03, 1.08E-05 to 1.45E-02, 2.16E-05 to 5.17E-02, 2.70E-05 to 1.39E-02, 4.00E-03 to 5.43E-02 and 4.70E-03 to 2.38E-02 mg/day respectively, while in case of children DIM ranged from 3.07E-04 to 1.13E-02, 8.16E-05 to 6.36E-03, 1.25E-05 to 2.28E-03, 1.25E-05 to 1.68E-02, 2.51E-05 to 6.01E-02, 3.14E-05 to 1.62E-02, 4.65E-03 to 1.25E-01 and 4.41E-03 to 2.77E-02 mg/day respectively as shown in Table 5. The daily intake of metals in Swabi for Pb, Cr, Cd, Ni, Zn, Cu, Fe and Mn for adults ranged from 3.72E-05 to 2.38E-03, 7.56E-05 to 1.80E-01, 1.08E-05 to 1.38E-03, 1.08E-05 to 1.01E-02, 1.62E-05 to 4.05E-02, 1.62E-05 to 1.05E-02, 2.53E-03 to 2.88E-02 and 2.07E-03 to 1.73E-02 mg/day respectively, while in case of children DIM ranged from 2.44E-04 to 8.77E-01, 8.79E-05 to 2.78E-03, 1.25E-05 to 1.61E-03, 1.25E-05 to 1.14E-01, 1.88E-05 to 4.71E-02, 1.88E-05 to 1.22E-02, 2.94E-03 to 3.36E-02 and 2.41E-03 to 1.98E-02 mg/day respectively as shown in Table 6. Randhawa *et al*. reported a high value of DIM for Pb (4.9E-2) and Cu (8.50E-2) as compared to the present value for Pb (5.23E-4) and Cu (2.24E-3) in the study areas of Multan, Pakistan [30]. Khan *et al*. investigated a low level of contamination due to clean water irrigation within the safe limit of DIM as that of the present study [31]. The present study of tubewell water irrigation posing no threat to human beings due to the consumption of vegetables.

**Table 6:** DIM and HRI for wastewater irrigated vegetables of district Swabi.

**Vegetables**			**Pb**	**Cr**	**Cd**	**Ni**	**Zn**	**Cu**	**Fe**	**Mn**
**Spinach**	Adult	DIM	5.51E-03	5.16E-03	6.21E-04	1.05E-02	8.71E-03	8.25E-03	6.93E-03	2.19E-02
		HRI	13.7E+00	3.44E-03	6.21E-01	5.28E-01	2.90E-02	2.06E-01	4.95E-02	6.66E-01
	Child	DIM	6.41E-03	6.01E-03	7.22E-04	1.22E-02	1.01E-02	9.59E-03	8.06E-03	2.55E-02
		HRI	16.0E+00	4.0E-03	7.22E-01	6.14E-01	3.37E-02	2.39E-01	5.76E-02	7.74E-01
**Cabbage**	Adult	DIM	9.79E-03	5.47E-03	1.96E-03	1.03E-02	7.86E-03	9.64E-03	1.04E-02	5.01E-03
		HRI	24.4E+00	3.65E-03	1.96E+00	5.16E-01	2.62E-02	2.41E-01	7.49E-02	1.51E-01
	Child	DIM	1.13E-02	6.36E-03	2.28E-03	1.20E-02	9.15E-03	1.12E-02	1.21E-02	5.82E-03
		HRI	28.4E+00	4.24E-03	2.28E+00	6.0E-01	3.05E-02	8.0E-02	8.71E-02	1.76E-01
**Cauliflower**	Adult	DIM	8.71E-03	9.18E-03	4.96E-04	9.02E-03	4.93E-03	9.56E-03	8.86E-03	9.18E-03
		HRI	21.7E+00	6.12E-03	4.96E-01	4.51E-01	1.64E-02	2.39E-01	6.33E-02	2.78E-01
	Child	DIM	1.01E-02	1.06E-02	5.77E-04	1.04E-02	5.73E-03	1.11E-02	1.03E-02	1.06E-02
		HRI	25.3E+00	7.11E-03	5.77E-01	5.24E-01	1.91E-02	2.78E-01	7.36E-02	3.23E-01
**Radish**	Adult	DIM	1.4203E-3	2.322E-4	1.89E-4	7.129E-4	8.101E-4	2.916E-4	6.8047E-3	3.796E-3
		HRI	3.55E-1	1.54E-4	1.89E-1	3.56E-2	2.70E-3	7.29E-3	4.86E-2	1.15E-1
	Child	DIM	1.6517E-3	2.701E-4	2.198E-4	8.29E-4	9.42E-4	3.391E-4	7.9131E-3	4.415E-3
		HRI	4.12E-1	1.80E-4	2.19E-1	4.14E-2	3.14E-3	8.47E-3	5.65E-2	1.33E-1
**Turnip**	Adult	DIM	3.15E-03	2.70E-03	1.32E-03	8.48E-03	7.78E-03	4.47E-03	4.0E-03	1.46E-02
		HRI	7.89E+00	1.80E-03	1.32E+00	4.24E-01	2.59E-02	1.11E-01	2.86E-02	4.44E-01
	Child	DIM	3.67E-03	3.14E-03	1.53E-03	9.86E-03	9.05E-03	5.19E-03	4.65E-03	1.70E-02
		HRI	9.18E+00	2.09E-03	1.53E+00	4.93E-01	3.01E-02	1.29E-01	3.32E-02	5.16E-01
**Tinda**	Adult	DIM	1.29E-03	1.35E-03	6.31E-04	8.94E-03	7.09E-03	3.15E-03	8.55E-03	1.0E-02
		HRI	3.24E+00	9.03E-04	6.31E-01	4.47E-01	2.36E-02	7.89E-02	6.11E-02	3.03E-01
	Child	DIM	1.50E-03	1.57E-03	7.34E-04	1.04E-02	8.25E-03	3.67E-03	9.95E-02	1.16E-02
		HRI	3.76E+00	1.05E-03	7.34E-01	5.20E-01	2.75E-02	9.18E-02	7.10E-02	3.53E-01
**Carrot**	Adult	DIM	4.39E-03	3.27E-03	6.96E-04	8.79E-03	4.70E-03	8.32E-03	1.42E-02	1.32E-02
		HRI	10.9E+00	2.18E-03	6.96E-01	4.39E-01	1.56E-02	2.08E-01	1.01E-01	4.02E-01
	Child	DIM	5.11E-03	3.81E-03	8.10E-04	1.02E-02	5.46E-03	9.68E-03	1.65E-02	1.54E-02
		HRI	12.7E+00	2.54E-03	8.10E-01	5.11E-01	1.82E-02	2.42E-01	1.18E-01	4.67E-01
**Lettuce**	Adult	DIM	2.77E-03	2.88E-03	1.63E-03	1.45E-02	7.86E-03	5.55E-03	1.01E-02	1.42E-02
		HRI	6.93E+00	1.92E-03	1.63E+00	7.25E-01	2.62E-02	1.38E-01	7.27E-02	4.32E-01
	Child	DIM	3.22E-03	3.35E-03	1.89E-03	1.68E-02	9.14E-03	6.45E-03	1.18E-02	1.65E-02
		HRI	8.06E+00	2.23E-03	1.89E+00	8.43E-01	3.04E-02	1.61E-01	8.45E-02	5.02E-01
**Colocasia**	Adult	DIM	1.40E-03	1.12E-03	7.61E-04	1.23E-02	3.93E-03	1.04E-02	6.32E-03	1.21E-02
		HRI	3.52E+00	7.52E-04	7.61E-01	6.17E-01	1.31E-02	2.60E-01	4.51E-02	3.69E-01
	Child	DIM	1.63E-03	1.31E-03	8.85E-04	1.43E-02	4.57E-03	1.21E-02	7.35E-03	1.41E-02
		HRI	4.09E+00	8.75E-04	8.85E-01	7.17E-01	1.52E-02	3.02E-01	5.25E-02	4.29E-01
**Vegetables**			**Pb**	**Cr**	**Cd**	**Cu**	**Zn**	**Ni**	**Fe**	**Mn**
**Bootlegourd**	Adult	DIM	3.78E-04	4.05E-04	2.16E-05	3.51E-03	1.11E-02	5.48E-03	1.14E-02	9.18E-03
		HRI	9.45E-01	2.70E-04	2.16E-02	1.75E-01	3.71E-02	1.37E-01	8.16E-02	2.78E-01
	Child	DIM	4.39E-04	4.71E-04	2.51E-05	4.08E-03	1.29E-02	6.39E-03	1.32E-02	1.06E-02
		HRI	1.09E+00	3.14E-04	2.51E-02	2.04E-01	4.32E-02	1.59E-01	9.49E-02	3.23E-01
**Tomato**	Adult	DIM	5.56E-04	5.29E-04	1.08E-05	1.08E-05	1.15E-02	1.31E-02	3.43E-02	4.70E-03
		HRI	1.39E+00	3.52E-04	1.08E-02	5.40E-04	3.85E-02	3.27E-01	2.45E-01	1.42E-01
	Child	DIM	6.46E-04	6.15E-04	1.25E-05	1.25E-05	1.34E-02	1.52E-02	3.99E-02	5.46E-03
		HRI	1.61E+00	4.10E-04	1.25E-02	6.25E-04	4.48E-02	3.81E-01	2.85E-01	1.65E-01
**Cucumber**	Adult	DIM	7.77E-04	6.53E-04	4.15E-04	7.56E-03	2.04E-02	6.24E-03	5.51E-02	8.25E-03
		HRI	1.94E+00	4.35E-04	4.15E-01	3.78E-01	6.81E-02	1.56E-01	3.94E-01	2.50E-01
	Child	DIM	9.04E-04	7.59E-04	4.83E-04	8.79E-03	2.37E-02	7.26E-03	6.41E-02	9.59E-03
		HRI	2.26E+00	5.06E-04	4.83E-01	4.39E-01	7.92E-02	1.81E-01	4.58E-01	2.90E-01
**Potato**	Adult	DIM	1.39E-03	3.40E-04	2.70E-04	1.62E-03	1.12E-02	4.40E-03	6.56E-03	9.72E-03
		HRI	3.48E+00	2.26E-04	2.70E-01	8.10E-02	3.75E-02	1.10E-01	4.69E-02	2.94E-01
	Child	DIM	1.62E-03	3.95E-04	3.14E-04	1.88E-03	1.30E-02	5.12E-03	7.63E-03	1.13E-02
		HRI	4.05E+00	2.63E-04	3.14E-01	9.42E-02	4.36E-02	1.28E-01	5.45E-02	3.42E-01
**Red pepper**	Adult	DIM	5.40E-04	5.40E-04	1.08E-05	1.56E-04	1.21E-02	1.39E-02	3.87E-02	1.35E-02
		HRI	1.35E+00	1.90E-04	1.08E-02	7.83E-03	4.05E-02	3.48E-01	2.76E-01	2.76E-01
	Child	DIM	6.28E-04	3.32E-04	1.26E-05	1.82E-04	1.41E-02	1.62E-02	4.50E-02	1.57E-02
		HRI	1.57E+00	2.21E-04	1.26E-02	9.10E-03	4.71E-02	4.05E-01	3.21E-01	4.75E-01
**Coriander**	Adult	DIM	5.77E-04	3.61E-04	8.10E-05	5.47E-03	1.35E-02	8.40E-03	5.43E-02	1.18E-02
		HRI	1.44E+00	2.41E-04	8.10E-02	2.73E-01	4.50E-02	2.10E-01	3.88E-01	3.60E-01
	Child	DIM	6.72E-04	4.20E-04	9.42E-05	6.36E-03	1.57E-02	9.77E-03	6.32E-02	1.38E-02
		HRI	1.68E+00	2.80E-04	9.42E-02	3.18E-01	5.23E-02	2.44E-01	4.51E-01	4.18E-01
**Bitter gourd**	Adult	DIM	5.56E-04	7.02E-05	1.62E-05	2.70E-05	2.16E-05	2.70E-05	1.22E-02	5.40E-03
		HRI	1.39E+00	4.68E-05	1.62E-02	1.35E-03	7.20E-05	6.75E-04	8.74E-02	1.63E-01
	Child	DIM	6.46E-04	8.16E-05	1.88E-05	3.14E-05	2.51E-05	3.14E-05	1.42E-02	6.28E-03
		HRI	1.61E+00	5.44E-05	1.88E-02	1.57E-03	8.36E-05	7.85E-04	1.01E-01	1.90E-01
**Green pepper**	Adult	DIM	4.69E-04	1.13E-04	1.51E-04	4.49E-03	5.17E-02	7.02E-03	5.13E-02	2.38E-02
		HRI	1.17E+00	7.56E-05	1.51E-01	2.24E-01	1.72E-01	1.75E-01	3.66E-01	7.22E-01
	Child	DIM	5.46E-04	1.31E-04	1.75E-04	5.23E-03	6.01E-02	8.16E-03	5.96E-02	2.77E-02
		HRI	1.36E+00	8.79E-05	1.75E-01	2.61E-01	2.0E-01	2.04E-01	4.26E-01	8.40E-01
**Brinjal**	Adult	DIM	5.23E-04	4.05E-04	1.02E-04	1.45E-03	1.05E-02	1.30E-02	3.78E-02	1.93E-02
		HRI	1.30E+00	2.70E-04	1.02E-01	7.26E-02	3.51E-02	3.26E-01	2.70E-01	5.86E-01
	Child	DIM	6.09E-04	4.71E-04	1.19E-04	1.68E-03	1.22E-02	1.51E-02	4.40E-02	2.25E-02
		HRI	1.52E+00	3.14E-04	4.93E-01	8.40E-02	4.08E-02	3.70E-01	3.14E-01	6.81E-01
**Vegetables**			**Pb**	**Cr**	**Cd**	**Cu**	**Zn**	**Ni**	**Fe**	**Mn**
**Pea**	Adult	DIM	2.38E-03	8.64E-04	1.20E-03	9.45E-03	1.27E-02	1.12E-02	1.22E-02	2.11E-02
		HRI	5.95E+00	5.76E-04	1.20E+00	4.72E-01	4.25E-02	5.62E-01	8.74E-02	6.40E-01
	Child	DIM	2.76E-03	1.0E-03	1.40E-03	1.09E-02	1.48E-02	1.30E-02	1.42E-02	2.45E-02
		HRI	6.92E+00	6.69E-04	1.40E+00	5.49E-01	4.95E-02	6.54E-01	1.01E-01	7.45E-01
**Pumpkin**	Adult	DIM	2.64E-04	7.07E-04	1.62E-05	4.67E-03	1.93E-02	9.35E-03	1.08E-02	1.14E-02
		HRI	6.61E-01	4.71E-04	1.62E-02	2.33E-01	6.45E-02	2.33E-01	7.71E-02	3.46E-01
	Child	DIM	3.07E-04	8.22E-04	1.88E-05	5.43E-03	2.25E-02	1.08E-02	1.25E-01	1.32E-02
		HRI	7.69E-01	5.48E-04	1.88E-02	2.71E-01	7.50E-02	2.72E-01	8.97E-02	4.02E-01
**Onion**	Adult	DIM	2.20E-03	9.01E-04	8.42E-04	8.45E-03	1.0E-02	3.72E-04	8.54E-03	6.92E-03
		HRI	5.50E+00	6.01E-04	8.42E-01	4.22E-01	3.35E-02	9.31E-03	6.10E-02	2.09E-01
	Child	DIM	2.56E-03	1.04E-03	9.79E-04	9.83E-03	1.17E-02	4.33E-04	9.94E-03	8.05E-03
		HRI	6.40E+00	6.99E-04	9.79E-01	4.91E-01	3.90E-02	1.08E-02	7.10E-02	2.44E-01
**Garlic**	Adult	DIM	2.74E-03	8.37E-04	1.12E-03	1.21E-02	1.84E-02	3.37E-03	1.51E-02	1.22E-02
		HRI	6.85E+00	5.58E-04	1.12E+00	6.07E-01	6.14E-02	8.43E-02	1.08E-01	3.70E-01
	Child	DIM	3.19E-03	9.73E-04	1.31E-03	1.41E-02	2.14E-02	3.92E-03	1.75E-02	1.42E-02
		HRI	7.97E+00	6.48E-04	1.31E+00	7.06E-01	7.15E-02	9.81E-02	1.25E-01	4.31E-01
**Green amaranth**	Adult	DIM	1.14E-03	4.96E-04	8.64E-05	1.26E-03	1.97E-02	5.84E-03	7.56E-03	1.25E-02
		HRI	2.86E+00	3.31E-04	8.64E-02	6.31E-02	6.57E-02	1.46E-01	5.40E-02	3.79E-01
	Child	DIM	1.33E-03	5.77E-04	1.04E-04	1.46E-03	2.29E-02	6.80E-03	8.79E-03	1.45E-02
		HRI	3.32E+00	3.85E-04	1.04E-01	7.34E-02	7.64E-02	1.70E-01	6.23E-02	4.40E-01
		HRI	2.85E+00	5.61E-04	1.82E-01	2.14E-01	6.13E-02	3.03E-01	1.42E-01	3.71E-01

To assess the health risk associated with the chemical contaminant, it is important to investigate the level of exposure and risk index. In the current study area, dietary vegetables grown were mostly used in the locality, for that reason the mean metal level was taken for HRI. The HRI in Swabi for Pb, Cr, Cd, Ni, Zn, Cu, Fe and Mn for adults ranged from 3.55E-01 to 24.4E+00, 4.68E-05 to 6.12E-03, 1.08E-02 to 1.96E+00, 5.40E-04 to 7.25E-01, 7.20E-05 to 1.72E-01, 6.75E-04 to 3.48E-01, 2.86E-02 to 3.94E-01 and 1.15E-01 to 7.22E-01 mg/day respectively, while in case of children, HRI ranged from 4.12E-01 to 28.4E+00, 5.44E-05 to 7.11E-03, 1.25E-02 to 2.28E+00, 6.25E-04 to 8.43E-01, 8.36E-05 to 2.01E-01, 7.85E-04 to 4.05E-01, 3.32E-02 to 4.58E-01 and 1.33E-01 to 8.40E-01 mg/day as shown in Table 6 respectively. The study reported a high value of HRI more than 1 for Pb in spinach, cabbage, cucumber, potato, red pepper, coriander, bitter gourd, pea, onion, garlic and green amaranth in Peshawar respectively. A high value of HRI was observed for Cd in spinach, cabbage, turnip, tinda, carrot, lettuce, colocasia, pea, onion and garlic. A high value of HRI was observed for Mn in green pepper while for Cu in tinda. In the case of Swabi, a high value of HRI was found for Pb in all vegetables while Cd showed contamination in cabbage, turnip, lettuce, pea and garlic respectively.

The HRI in freshwater irrigated vegetables of Swabi for Pb, Cr, Cd, Ni, Zn, Cu, Fe and Mn for adults ranged from 1.56E-01 to 5.96E+00, 5.04E-05 to 1.20E-01, 1.08E-02 to 1.38E+00, 5.40E-04 to 5.09E-01, 5.40E-04 to 1.35E-01, 4.05E-04 to 2.63E-01, 2.80E-02 to 2.07E-01 and 6.28E-02 to 5.25E-01 mg/day respectively, while in case of children HRI ranged from 1.82E-01 to 6.93E+00, 5.86E-05 to 4.32E-02, 1.25E-02 to 1.61E+00, 6.25E-04 to 5.70E+00, 6.26E-05 to 7.67E-02, 4.70E-04 to 3.06E-01, 2.10E-02 to 2.40E-01 and 7.30E-02 to 6.11E-01 mg/day respectively as shown in Table 7. In the case of Swabi, HRI for Pb was found higher in all vegetables while Cd showed high value (HRI > 1) in turnip and lettuce and Ni showed contamination in brinjal. Zhuang*et al*. found HRI for Cd and Pb exceeding safe limits in vegetables irrigated with polluted water in Guangdong, China [32]. Cui *et al*. indicated that Cd and Pb were the main threat posing elements in China which was also in close agreement with the current work [33].

**Table 7:** DIM and HRI for fresh water irrigated vegetables of district Swabi.

**Vegetables**			**Pb**	**Cr**	**Cd**	**Cu**	**Zn**	**Ni**	**Fe**	**Mn**
**Spinach**	Adult	DIM	2.31E-03	2.34E-03	5.07E-04	9.64E-03	8.32E-03	8.10E-03	5.55E-03	1.73E-02
		HRI	5.77E+00	1.56E-03	5.07E-01	4.82E-01	2.77E-02	2.02E-01	3.96E-02	5.25E-01
	Child	DIM	2.68E-03	2.72E-03	5.90E-04	1.12E-02	9.68E-03	9.42E-03	6.45E-03	2.01E-02
		HRI	6.71E+00	1.81E-03	5.90E-01	5.60E-01	3.22E-02	2.35E-01	4.61E-02	6.11E-01
**Cabbage**	Adult	DIM	2.31E-03	2.0E-03	6.31E-04	8.02E-03	6.86E-03	7.63E-03	8.64E-03	4.23E-03
		HRI	5.77E+00	1.33E-03	6.31E-01	4.01E-01	2.28E-02	1.90E-01	6.17E-02	1.28E-01
	Child	DIM	2.68E-03	2.32E-03	7.34E-04	9.31E-03	7.98E-03	8.87E-03	1.0E-02	4.92E-03
		HRI	6.71E+00	1.55E-03	7.34E-01	4.65E-01	2.66E-02	2.21E-01	7.17E-02	1.49E-01
**Cauliflower**	Adult	DIM	1.89E-03	2.39E-03	2.97E-04	7.56E-03	3.08E-03	5.08E-03	7.24E-03	8.48E-03
		HRI	4.72E+00	1.59E-03	2.97E-01	3.78E-01	1.02E-02	1.27E-01	5.17E-02	2.57E-01
	Child	DIM	2.19E-03	2.78E-03	3.45E-04	8.79E-03	3.58E-03	5.91E-03	8.42E-03	9.86E-03
		HRI	5.49E+00	1.85E-03	3.45E-01	4.39E-01	1.19E-02	1.47E-01	6.01E-02	2.98E-01
**Radish**	Adult	DIM	6.265E-4	1.134E-4	1.35E-4	2.484E-4	5.887E-4	1.566E-4	2.5329E-3	2.073E-3
		HRI	1.56E-1	7.56E-5	1.35E-1	1.24E-2	1.96E-3	3.91E-3	1.80E-2	6.28E-2
	Child	DIM	7.285E-4	1.319E-4	1.57E-4	2.889E-4	6.845E-4	1.821E-4	2.9454E-3	2.411E-3
		HRI	1.82E-1	8.79E-5	1.57E-1	1.44E-2	2.28E-3	4.55E-3	2.10E-2	7.30E-2
**Turnip**	Adult	DIM	1.12E-03	1.13E-03	1.15E-03	6.24E-03	6.01E-03	2.31E-03	3.93E-03	1.15E-02
		HRI	2.80E+00	7.56E-04	1.15E+00	3.12E-01	2.0E-02	5.77E-02	2.80E-02	3.50E-01
	Child	DIM	1.30E-03	1.31E-03	1.33E-03	7.26E-03	6.99E-03	2.68E-03	4.57E-03	1.34E-02
		HRI	3.26E+00	8.79E-04	1.33E+00	3.63E-01	2.33E-02	6.71E-02	3.26E-02	4.07E-01
**Tinda**	Adult	DIM	8.20E-04	1.80E-01	6.15E-04	6.81E-03	6.24E-03	2.61E-03	6.24E-03	7.71E-03
		HRI	2.05E+00	1.20E-01	6.15E-01	3.40E-01	2.08E-02	6.54E-02	4.46E-02	2.33E-01
	Child	DIM	9.54E-04	1.51E-03	7.15E-04	7.91E-03	7.26E-03	3.04E-03	7.26E-03	8.96E-03
		HRI	2.38E+00	1.01E-03	7.15E-01	3.95E-01	2.42E-02	7.61E-02	5.18E-02	2.71E-01
**Carrot**	Adult	DIM	1.96E-03	1.69E-03	7.39E-04	8.55E-03	4.23E-03	7.02E-03	9.79E-03	8.40E-03
		HRI	4.91E+00	1.13E-03	7.39E-01	4.27E-01	1.41E-02	1.75E-01	6.99E-02	2.54E-01
	Child	DIM	2.28E-03	1.97E-03	8.60E-04	9.95E-03	4.92E-03	8.16E-03	1.13E-02	9.77E-03
		HRI	5.71E+00	1.31E-03	8.60E-01	4.97E-01	1.64E-02	2.04E-01	8.13E-02	2.96E-01
**Lettuce**	Adult	DIM	2.38E-03	1.73E-03	1.38E-03	9.94E-03	6.55E-03	2.85E-03	4.77E-03	9.87E-03
		HRI	5.96E+00	1.15E-03	1.38E+00	4.97E-01	2.18E-02	7.12E-02	3.41E-02	2.99E-01
	Child	DIM	2.77E-03	2.01E-03	1.61E-03	1.15E-02	7.62E-03	3.31E-03	5.55E-03	1.14E-02
		HRI	6.93E+00	1.34E-03	1.61E+00	5.78E-01	2.54E-02	8.28E-02	3.96E-02	3.47E-01
**Colocasia**	Adult	DIM	1.13E-03	1.06E-03	7.29E-04	1.01E-02	3.24E-03	6.01E-03	3.93E-03	8.55E-03
		HRI	2.84E+00	7.09E-04	7.29E-01	5.09E-01	1.08E-02	1.50E-01	2.80E-02	2.59E-01
	Child	DIM	1.32E-03	1.23E-03	8.47E-04	1.18E-02	3.76E-03	6.99E-04	4.57E-03	9.95E-03
		HRI	3.31E+00	8.24E-04	8.47E-01	3.77E-01	1.25E-02	1.74E-01	3.26E-02	3.01E-01
**Vegetables**			**Pb**	**Cr**	**Cd**	**Cu**	**Zn**	**Ni**	**Fe**	**Mn**
**Bootlegourd**	Adult	DIM	2.86E-04	2.70E-04	1.08E-05	2.06E-03	7.10E-03	4.22E-03	8.81E-03	8.64E-03
		HRI	7.15E-01	1.80E-04	1.08E-02	1.03E-01	2.36E-02	1.05E-01	6.29E-02	2.61E-01
	Child	DIM	3.32E-04	3.14E-04	1.26E-05	2.40E-03	8.26E-03	4.91E-03	1.05E-02	1.0E-02
		HRI	8.32E-01	2.09E-04	1.26E-02	1.20E-01	2.75E-02	1.22E-01	7.32E-02	3.04E-01
**Tomato**	Adult	DIM	4.75E-04	3.88E-04	1.08E-05	1.08E-05	9.94E-03	8.48E-03	1.77E-02	4.0E-03
		HRI	1.18E+00	2.59E-04	1.08E-02	5.40E-04	3.31E-02	2.12E-01	1.26E-01	1.21E-01
	Child	DIM	5.52E-04	4.52E-04	1.25E-05	1.25E-05	1.15E-02	9.86E-03	2.06E-02	4.65E-03
		HRI	1.38E+00	3.01E-04	1.25E-02	6.25E-04	3.85E-02	2.46E-01	1.47E-01	1.41E-01
**Cucumber**	Adult	DIM	6.48E-04	3.51E-04	1.99E-04	6.63E-03	1.62E-02	4.0E-03	2.77E-02	6.93E-03
		HRI	1.62E+00	2.34E-04	1.99E-01	3.31E-01	5.40E-02	1.0E-01	1.98E-01	2.10E-01
	Child	DIM	7.53E-04	4.08E-04	2.32E-04	7.71E-03	1.88E-02	4.65E-03	3.22E-02	8.09E-03
		HRI	1.88E+00	2.72E-04	2.32E-01	3.85E-01	6.28E-02	1.16E-01	2.30E-01	2.44E-01
**Potato**	Adult	DIM	9.93E-04	3.18E-04	2.21E-04	1.48E-03	1.08E-02	4.40E-03	6.38E-03	9.45E-03
		HRI	2.48E+00	2.12E-04	2.21E-01	7.42E-02	3.60E-02	1.10E-01	4.56E-02	2.86E-01
	Child	DIM	1.15E-03	3.70E-04	2.57E-04	1.72E-03	1.25E-02	5.12E-03	7.42E-03	1.09E-02
		HRI	2.88E+00	2.47E-04	2.57E-01	8.63E-02	4.18E-02	1.28E-01	5.30E-02	3.33E-01
**Red pepper**	Adult	DIM	4.32E-04	2.37E-04	1.62E-05	1.13E-04	1.16E-02	1.05E-02	2.89E-02	9.99E-03
		HRI	1.08E+00	1.58E-04	1.62E-02	5.67E-03	3.87E-02	2.63E-01	2.07E-01	3.02E-01
	Child	DIM	5.02E-04	2.76E-04	1.88E-05	1.31E-04	1.35E-02	1.22E-02	3.36E-02	1.16E-02
		HRI	1.25E+00	1.84E-04	1.88E-02	6.59E-03	4.50E-02	3.06E-01	2.40E-01	3.52E-01
**Coriander**	Adult	DIM	3.88E-04	2.53E-04	4.32E-05	2.46E-03	1.11E-02	6.93E-03	2.73E-02	9.79E-03
		HRI	9.72E-01	1.69E-04	4.32E-02	1.23E-01	3.70E-02	1.73E-01	1.95E-01	2.96E-01
	Child	DIM	4.52E-04	4.32E-04	5.02E-05	2.87E-03	1.29E-02	8.06E-03	3.18E-02	1.13E-02
		HRI	1.13E+00	4.32E-02	5.02E-02	1.43E-01	4.30E-02	2.01E-01	2.27E-01	3.45E-01
**Bitter gourd**	Adult	DIM	3.51E-04	1.08E-04	1.08E-05	1.62E-05	1.62E-05	1.62E-05	1.08E-02	3.78E-03
		HRI	8.77E-01	7.20E-05	1.08E-02	8.10E-04	5.40E-04	4.05E-04	7.77E-02	1.14E-01
	Child	DIM	4.08E-04	1.25E-04	1.25E-05	1.88E-05	1.88E-05	1.88E-05	1.26E-02	4.40E-03
		HRI	1.02E+00	8.37E-05	1.25E-02	9.40E-04	6.26E-05	4.70E-04	9.04E-02	1.33E-01
**Green pepper**	Adult	DIM	3.24E-04	7.56E-05	5.94E-05	3.68E-03	4.05E-02	5.94E-03	2.88E-02	1.70E-02
		HRI	8.10E-01	5.04E-05	5.94E-02	1.84E-01	1.35E-01	1.48E-01	2.05E-01	5.18E-01
	Child	DIM	3.76E-04	8.79E-05	6.91E-05	4.28E-03	4.71E-02	6.90E-03	3.34E-02	1.98E-02
		HRI	9.42E-01	5.86E-05	6.91E-02	2.14E-01	1.57E-01	1.72E-01	2.39E-01	6.02E-01
**Brinjal**	Adult	DIM	3.72E-05	3.99E-04	7.56E-05	1.25E-03	7.83E-03	9.72E-03	2.65E-02	1.57E-02
		HRI	9.31E-01	2.66E-04	7.56E-02	6.29E-02	2.61E-02	2.43E-01	1.89E-01	4.77E-01
	Child	DIM	4.33E-04	4.64E-04	8.79E-05	1.14E-01	9.10E-03	1.13E-02	3.08E-02	1.83E-02
		HRI	1.08E+00	3.09E-04	8.79E-02	5.7E+00	3.03E-02	2.82E-01	2.20E-01	5.54E-01
**Vegetables**			**Pb**	**Cr**	**Cd**	**Cu**	**Zn**	**Ni**	**Fe**	**Mn**
**Pea**	Adult	DIM	9.88E-04	6.37E-04	2.97E-04	9.89E-03	1.0E-02	7.18E-04	8.09E-03	9.99E-03
		HRI	2.47E+00	4.24E-04	2.97E-01	4.94E-01	3.35E-02	1.79E-02	5.72E-02	3.02E-01
	Child	DIM	1.14E-03	7.41E-04	3.45E-04	1.15E-02	1.17E-02	8.35E-04	9.31E-03	1.16E-02
		HRI	2.87E+00	4.94E-04	3.45E-01	5.15E-01	3.90E-02	2.08E-02	6.65E-02	3.52E-01
**Pumpkin**	Adult	DIM	2.10E-04	3.67E-04	1.08E-05	2.60E-03	1.57E-02	8.64E-03	1.06E-02	1.01E-02
		HRI	5.26E-01	2.44E-04	1.08E-02	1.30E-01	5.24E-02	2.16E-01	7.58E-02	3.08E-01
	Child	DIM	2.44E-04	4.27E-04	1.25E-05	3.03E-03	1.83E-02	1.00E-02	1.23E-02	1.18E-02
		HRI	6.12E-01	2.84E-04	1.25E-02	1.51E-01	6.10E-02	2.51E-01	8.81E-02	3.58E-01
**Onion**	Adult	DIM	6.80E-04	3.67E-04	3.29E-04	6.56E-03	7.64E-03	3.02E-04	6.11E-03	5.48E-03
		HRI	1.70E+00	2.44E-04	3.29E-01	3.28E-01	2.54E-02	7.56E-03	4.37E-02	1.66E-01
	Child	DIM	7.91E-04	4.27E-04	3.83E-04	7.63E-03	8.89E-03	3.51E-04	7.11E-03	6.38E-03
		HRI	1.97E+00	2.84E-04	3.83E-01	3.81E-01	2.96E-02	8.79E-03	5.08E-02	1.93E-01
**Garlic**	Adult	DIM	1.26E-03	5.13E-04	6.69E-04	7.56E-03	1.74E-02	2.24E-03	1.21E-02	9.08E-03
		HRI	3.17E+00	3.42E-04	6.69E-01	3.78E-01	5.83E-02	5.61E-02	8.67E-02	2.75E-01
	Child	DIM	1.47E-03	5.96E-04	7.78E-04	8.79E-03	2.03E-02	2.61E-03	1.41E-02	1.05E-02
		HRI	3.46E+00	3.97E-04	7.78E-01	4.39E-01	6.78E-02	6.53E-02	1.00E-01	3.20E-01
**Green amaranth**	Adult	DIM	8.04E-04	4.91E-04	7.56E-05	9.18E-04	1.98E-02	4.49E-03	7.29E-03	9.90E-03
		HRI	2.01E+00	3.27E-04	7.56E-02	4.59E-02	6.60E-02	1.12E-01	5.20E-02	3.30E-01
	Child	DIM	9.35E-04	5.71E-04	8.79E-05	1.06E-03	2.30E-02	5.23E-03	8.47E-03	1.15E-02
		HRI	2.33E+00	3.80E-04	8.79E-02	5.33E-02	7.67E-02	1.30E-01	6.05E-02	3.48E-01

### Enrichment factor

Enrichment factor (EF) is the investigation of the transfer of heavy metals from soil to vegetables and to show variation in the metal accumulation in vegetables among various areas. Lower values of enrichment factor may be due to high retention of metals in the soil and poor translocation in the vegetables. The enrichment factor of metals in Swabi for Pb, Cr, Cd, Ni, Zn, Cu, Fe and Mn ranged from 0.65 to 2.61, 0.29 to 1.47, 0.14 to 1.32, 0.29 to 2.05, 0.16 to 0.90, 0.49 to 1.18, 0.64 to 1.37 and 0.56 to 1.12 respectively as shown in Table 8. In the case of sector-S, EF of Pb was high in cabbage (2.40), cauliflower (2.61), Cr in radish (2.64), cauliflower (1.47), Ni (2.33) and Fe (2.29) in radish, respectively. Fytianas *et al*. investigated the high value of EF for Cd in leafy vegetables [34]. Sridhara *et al*. in one study also analyzed the higher EF value of heavy metals in leafy vegetables [35].

**Table 8:** Enrichment factor of heavy metals in vegetables of district Swabi.

Vegetables	Pb	Cr	Cd	Ni	Zn	Cu	Fe	Mn
**Spinach**	1.35	0.84	0.37	0.92	0.74	0.76	1.07	1.19
**Cabbage**	2.40	1.05	0.96	1.08	0.84	0.95	1.02	1.12
**Cauliflower**	2.61	1.47	0.51	1	1.16	1.42	1.05	1.02
**Radish**	1.21	2.64	0.93	2.33	1	0.82	2.29	1.78
**Turnip**	1.58	0.91	0.35	1.14	0.92	1.48	0.88	1.19
**Tinda**	0.88	0.39	0.31	1.10	0.81	0.92	1.18	1.23
**Carrot**	1.26	0.74	0.29	0.86	0.80	0.89	1.25	1.49
**Lettuce**	0.65	0.64	0.36	1.22	0.87	1.49	1.85	1.36
**Colocasia**	0.69	0.41	0.32	1.01	0.87	1.29	1.40	1.34
**Bootle gourd**	0.75	0.57	0.60	1.45	1.13	0.97	1.11	1
**Tomato**	0.65	0.52	0.20	0.38	0.84	1.16	1.66	1.12
**Cucumber**	0.66	0.71	0.64	0.95	0.89	1.17	1.70	1.12
**Potato**	0.78	0.40	0.37	0.93	0.75	0.75	0.88	0.97
**Red pepper**	0.72	0.45	0.14	1.16	0.75	0.99	1.14	1.27
**Coriander**	0.87	0.54	0.55	1.89	0.90	0.91	1.68	1.14
**Bitter gourd**	0.90	0.25	0.46	1	1	1	1	1.35
**Green pepper**	0.84	0.57	0.77	1.03	0.91	0.88	1.09	1.32
**Brinjal**	0.75	0.38	0.40	1	0.98	1	1.22	1.16
**Pea**	1.35	0.51	1.32	0.95	0.91	1.29	1.31	2
**Pumpkin**	0.66	0.73	0.40	1.51	0.87	0.81	0.87	1.06
**Onion**	1.82	0.94	0.78	1.08	0.95	0.92	1.20	1.20
**Garlic**	1.22	0.62	0.52	1.35	0.76	1.16	1.06	1.27
**Green amaranth**	0.79	0.38	0.34	1.19	0.71	0.98	0.89	1.19

## Conclusion

The concentration of Cr in wastewater and soil was found higher than the permissible limit of WHO (1996).Mean concentration of Pb (14.210 mg/kg) was found higher in cabbage, Cr (12.925 mg/kg) in cauliflower, Cd (3.110 mg/kg) in lettuce, Ni (22.70 mg/kg) in colocasia, Zn (94.81 mg/kg) and Fe (90.91 mg/kg) in green pepper, Cu (24.23 mg/kg) in red pepper and Mn (39.89 mg/kg) in spinach respectively. The transfer factor of Cr and Cd was found to be 2.82 and 6.42 respectively. HRI for Pb in cabbage, 24.4E+00 for adult, 28.4E+00 for children and Cd, 1.96E+00 for adult and 2.28E+00 for children respectively. HRI for Pb in lettuce showed 5.96E+00 for adults, 6.96E+00 for children and Cd, 1.38E+00 for adults and 1.61E+00 for children respectively. Enrichment factor (EF) of Pb, Cr and Ni was found high in Swabi in red pepper, onion, cabbage, cauliflower, spinach, garlic and radish. Fresh dietary vegetables cultivated using wastewater showed heavy metal accumulation especially Pb, Cr, Cd, Ni which crossed the safe limits of WHO (1996). The study further suggested that even a low concentration of heavy metals in wastewater raises a threat to human life by accumulation over a longer time. The results obtained here demand proper legislation, urgent implementation of appropriate safety measures and consistent monitoring of heavy metals released into water and soil. Industrial and municipal effluents must be treated before released into sewage water, to combat soil and vegetable contamination.Based on the findings of this study, there would be a significant risk to the consumers associated with consumptions of vegetables being cultivated in Gadoon Industrial Estate area of district Swabi. Therefore, strict regulatory control measures are highly recommended on the safety of vegetables originated from the study area.

## Supporting information

S1 Table List of dietary vegetables used in this study. (DOCX)
